# Semen Analysis of Total Motile Sperm Count Based on the 1999 and 2010 WHO Criteria

**DOI:** 10.5935/1518-0557.20210066

**Published:** 2022

**Authors:** Patrícia de Moraes De Zorzi, Ana Paula de Souza Kussler, Anita Mylius Pimentel, Edison Capp, Helena von Eye Corleta

**Affiliations:** 1 Programa de Pós-Graduação em Ciências da Saúde: Ginecologia e Obstetrícia, Medicine School, Universidade Federal do Rio Grande do Sul, Porto Alegre, RS, Brazil; 2 Generar - Human Reproduction, Porto Alegre, RS, Brazil; 3 Department of Obstetrics and Gynecology, Medicine School, Universidade Federal do Rio Grande do Sul, Porto Alegre, RS, Brazil

**Keywords:** male fertility, semen analysis, seminal parameters, sperm function

## Abstract

**Objective:**

Approximately 15% of the couples suffer from infertility. Half of the cases of infertility are due to male factors. Several sperm function tests have been proposed to evaluate male fertility, but sperm analysis is still the first and most important diagnostic test for male infertility. The prognostic value of semen characteristics such as concentration, morphology and motility markers are often confused with male infertility. Evaluation of seminal parameters and classification for normality remains a frequent topic of discussion.

**Methods:**

This study evaluated 477 semen samples from men undergoing investigation or infertility treatment between 2011 and 2015.

**Results:**

The spermograms of 401 patients were deemed abnormal based on the 1999 World Health Organization (WHO) criteria; the number changed to 223 when the spermograms were assessed based on the 2010 WHO criteria and to 200 when Total Motile Sperm Count (TMSC) was used as the criterion. Sperm morphology was the item in the criteria that most significantly changed spermogram classification. Normality parameters became less rigid from 1999 to 2010, thereby significantly changing the proportion of individuals no longer described as infertile/subfertile.

**Conclusions:**

The classification based on TMSC could not differentiate between fertile and infertile subjects for not taking sperm morphology into account. Nevertheless, it may be helpful in cases where intrauterine insemination is indicated.

## INTRODUCTION

Approximately 15% of the couples suffer from infertility. Half of the cases of infertility are due to male factors (Tharakan *et al*., 2021). Several sperm function tests have been proposed to evaluate male fertility, but spermograms are the main diagnostic tool for male infertility (Talwar & Hayatnagarkar, 2015; Zhang *et al*., 2014).

Semen analysis is extremely important in the investigation of infertile couples and in the determination of a couple's ability to become pregnant. Before the publication of the World Health Organization (WHO) Manual in 1999, laboratories used different methods to obtain and analyze data and adopted diverse definitions for male fertility. This produced error in the identification of normal range values and led to the categorization of fertile men as infertile, when the ranges used to describe normality were too high and unrealistic, or infertile men as fertile, when the ranges were lower than what was needed to produce pregnancy. On the other hand, the population of men studied for the 2010 WHO Manual comprised individuals without proven paternity, patients attending human reproduction clinics seeking treatment, semen donors, and vasectomy candidates. In the last two groups of men, the first may be fertile because they have normal values and the second group is very likely to be fertile, although there is no data on the time it took for their partners to become pregnant (Vieira, 2013). Routine semen analysis alone has its limitations, since it does not take sperm dysfunctions such as immature chromatin or sperm DNA damage into consideration (Esteves *et al*., 2012).

Semen parameter evaluation, patient classification, and the definition of what constitutes normal range values are topics for discussion. In 1980, the first of five issues of the WHO Laboratory Manual for the Examination of Human Semen was published. The negative point of this first classification is that it was not validated by prospective studies (Catanzariti, 2013).

In 1999, the WHO described normal semen parameters based only on the study of fertile couples. This classification was based on data coming from various laboratories using different methodologies, and analyzed a number of populations without a standardized definition for fertile populations (Cooper *et al*., 2010).

In 2010, the WHO published more stringent guidelines, based on men who had naturally conceived children, a fact that does not necessarily imply that men with lower semen parameters are infertile (Hamilton *et al*., 2015). The new cutoff points were defined based on a study that included 1,953 men from various countries, whose wives became pregnant within less than a year. Values below the 5^th^ percentile of this group were considered abnormal. Normality was assigned to individuals with a Kruger score of 4% or higher. In addition, sperm motility classification was no longer used to separate sperm into grades a, b, c or d; instead, sperm was rated as having progressive motility, non-progressive motility, or immotile (WHO). Another classification studied is based on the Total Motile Sperm Count (TMSC). The result is obtained by multiplying the ejaculate volume by sperm concentration in milliliters and the proportion of motile sperm (a+b) divided by 100%, without taking into account the morphology or the performed seminal preprocessing (Ayala *et al*., 1996).

Therefore, the objective of this study was to evaluate and compare the influence of different semen classifications (1999 and 2010 WHO criteria; TMSC) on the diagnosis of male infertility.

## MATERIAL AND METHODS

This longitudinal retrospective study reviewed patient charts and looked into the characteristics of 477 male patients treated or tested for infertility between 2011 and 2015 at a private assisted reproduction clinic in Porto Alegre (Generar Human Reproduction). All patients in the period were enrolled (n=477). The Ethics Committee of the Hospital das Clínicas of Porto Alegre approved this study and awarded it certificate no. 20 16-0524. The collected data included age, use of medications, comorbidities, body mass index (BMI), days of abstinence, volume, concentration, motility, morphology (according to Tygerberg), round cells, leukocytes, vitality, and TMSC calculation. A single embryologist performed all semen evaluations.

Statistical analyses were performed on software package SPSS version 21.0, with the significance level set at 5% (*p*≤0.05). Quantitative variables expressed as means and standard error or as medians and interquartile ranges. Categorical variables were described with absolute and relative frequencies. Student's t-test was used to compare between means. Proportions were compared with Pearson's chi-squared test or Fisher's exact test. McNemar's test was used to compare between the alterations resulting from the use of the 1999 and 2010 WHO criteria.

## RESULTS

Semen samples of 477 patients aged 37 years on average were analyzed. Approximately 21% were obese and 10% smoked. More than 25% reported having comorbidities; 1% reported prior cancer treatment; 4.5% said they had taken psychoactive drugs; 5% had hypertension; 1.3% had insulin resistance; and 2.5% reported dyslipidemia.

The data on semen samples is shown in Table 1. The mean period of sexual abstinence before collection of semen was 3.65±1.77 days.

**Table 1.** Data from semen samples.

Variables	Data
Days of abstinence*	3.65±1.77
Volume (mL) *	2.84±1.43
Concentration (x106)#	32 (8 – 62)
Motility a+ b (%)*	38.6±17.5
Round cells (x106)#	2.6 (1.2 – 4.9)
Leukocytes (x106)#	0.8 (0.4 – 1.2)
Vitality (%)*	58.4±15.8
Normal morphology (%)#	10 (6 – 15)
TMSC (x106)#	28.9 (5.1 – 73.7)

* mean ± standard deviation;

# median (percentile 25-75).

TMSC: Total Motile Sperm Count

Significant changes were observed in almost every parameter when the 1999 and 2010 WHO criteria were compared, with the exception of total concentration. Of the 477 samples analyzed, 293 (61.4%) had at least two alterations according to the 1999 criteria; the number dropped to 112 (23.5%) when the samples were analyzed vis-à-vis the 2010 criteria.

Considering absolute and relative differences, the three parameters for which most alterations were found based on the 2010 criteria were morphology, vitality, and motility a+b (Table 2). Figure 1 illustrates these differences, with morphology showing as the parameter with most alterations according to the 1999 criteria that were rated as normal based on the 2010 criteria. Table 2 confirms this finding, as 85.1% of the samples did not show any alteration in morphology when they were classified based on the 2010 WHO criteria. When semen samples were analyzed based on the three classifications studied, 401 (84.1%) had alterations by the 1999 WHO criteria, 223 (46.8%) by the 2010 WHO criteria, and 200 (41.9%) had alterations based on TMSC (Table 3).

**Table 2.** Differences in parameter alterations based on the 1999 and 2010 WHO classifications.

Alterations	WHO		Absolute Difference (%)	Relative Difference (%)	*p*
	1999 n=477 (%)	2010 n=477 (%)			
Total concentration	163 (34.2)	162 (34.0)	0.2	0.6	1.000
Concentration/ml	170 (35.6)	146 (30.6)	5.0	14.0	<0.001
Motility a + b	310 (65.0)	151 (31.7)	33.3	51.2	<0.001
Morphology	335 (70.2)	50 (10.5)	59.7	85.0	<0.001
Vitality	400 (87.9)	175 (38.5)	49.4	56.2	<0.001
With at least 1 abnormal parameter*	401 (84.1)	223 (46.8)	37.3	44.4	<0.001
With at least 2 abnormal parameters*	293 (61.4)	112 (23.5)	37.9	61.7	<0.001

* The patient had alterations in any of the four parameters: total concentration, concentration/ml, motility and morphology.

WHO: World Health Organization.

**Table 3.** Alterations in 477 samples analyzed based on the 1999 and 2010 WHO classifications.

Variables	N=477	%
1999 WHO classification Total concentration < 40 million Concentration/ml < 20 x 106 Motility a + b < 50% Morphology < 14% With alterations – 4 general criteria* With at least 2 alterations	163 170 310 335 401 293	34.2 35.6 65.0 70.2 84.1 61.4
2010 WHO classification Total concentration < 39 million Concentration/ml < 15 x 10^6^ Motility a + b < 32% Morphology < 4% With at least 1 abnormal parameter* With at least 2 abnormal parameters*	162 146 151 50 223 112	34.0 30.6 31.7 10.5 46.8 23.5
TMSC (x10^6^) < 20 ≥ 20	200 277	41.9 58.1

* The patient had alteration in any of the four parameters (total concentration, concentration ml, motility and morphology).

TMSC: Total Motile Sperm Count; WHO: World Health Organization

**Figure 1:** Number of patients with alterations in sperm parameters according to the 1999 and 2010 WHO criteria WHO: World Health Organization.

When at least two of the clinically relevant semen parameters (total concentration, concentration per ml, motility and morphology) were altered, the number of samples considered abnormal decreased to 61.4% based on the 1999 WHO criteria and to 23.5% based on the 2010 WHO criteria (Table 3).

The analysis of the associations between normal (≥ 20 million) and altered samples (< 20 million) based on TMSC and the 1999 and 2010 WHO classifications are presented in Table 4. There was a significant association in all parameters. Of the 200 samples considered altered based on TMSC, 192 (96%) had at least two alterations based on the 1999 WHO criteria, compared with 108 (54%) according to the 2010 WHO classification. On the other hand, of the 277 samples considered normal by TMSC, 101 (36.5%) had more than two alterations based on the 1999 WHO criteria and only four (1.4%) had more than two alterations according to the 2010 WHO criteria.

**Table 4.** Association between TMSC and alterations in the 1999 and 2010 WHO classifications.

Variables	TMSC (x106)		*P*
	< 20 (n=200)	≥ 20 (n=277)	
1999 WHO Classification Total concentration < 40 million Concentration/ ml < 20 x 10^6^ Motility a + b < 50% Morphology < 14% With alterations - 4 general criteria* With at least 2 alterations	161 (80.5) 154 (77.0) 178 (89.0) 177 (88.5) 200 (100) 192 (96.0)	2 (0.7) 16 (5.8) 132 (47.7) 158 (57.0) 201 (72.6) 101 (36.5)	<0.001 <0.001 <0.001 <0.001 <0.001 <0.001
2010 WHO Classification Total concentration < 39 million Concentration/ ml < 15 x 10^6^ Motility a + b < 32% Morphology < 4% With at least 1 abnormal parameter* With at least 2 abnormal parameters*	160 (80.0) 140 (70.0) 129 (64.5) 46 (23.0) 193 (96.5) 108 (54.0)	2 (0.7) 6 (2.2) 22 (7.9) 4 (1.4) 30 (10.8) 4 (1.4)	<0.001 <0.001 <0.001 <0.001 <0.001 <0.001

* The patient had alterations in any of the four parameters: total concentration, concentration/ ml, motility and morphology

TMSC: Total Motile Sperm Count; WHO: World Health Organization.

Patients with motility alterations based on the 1999 and 2010 WHO criteria were significantly older and presented no association with TMSC. Based on the 1999 WHO criteria, men with motility disorders had significantly more days of abstinence (Table 5) without associations with TMSC or the 2010 WHO criteria.

**Table 5.** Significant associations between motility, morphology, volume, vitality and general (at least one criteria) alterations.

Variables	Motility a + b – 1999		*p*	Motility a + b – 2010		*P*
	< 50%	≥ 50%		< 32%	≥ 32%	
Age (years) ^#^	37.6±6.8	35.8±6.1	0.005	38.0±6.6	36.5±6.6	0.019^§^
Days of abstinence ^#^	3.76±2.02	3.45±1.15	0.035	3.70±2.32	3.63±1.45	0.691^§^
	Morphology (%) – 1999		*p*	Morphology (%) - 2010		*p*
	< 14	≥ 14		< 4	≥ 4	
Smoking - n (%)	45 (10.1)	0 (0.0)	1.000	9 (20.5)	36 (8.9)	0.029^†^
Presence of comorbidity - n(%)	82 (26.0)	33 (25.4)	0.982	21 (44.7)	94 (23.6)	0.003^†^
	Volume (ml) – 1999		*p*	Volume (ml) – 2010		*p*
	<2	≥ 2		<1.5	≥ 1.5	
Hypertension - n (%)	11 (9.5)	13 (3.6)	0.023	5 (8.3)	19 (4.6)	0.208^†^
Days of abstinence^#^	3.37±1.49	3.74±1.84	0.049	3.60±1.78	3.66±1.77	0.825^§^
	Vitality (%) – 1999		*p*	Vitality (%) – 2010		*p*
	<75	≥ 75		<58	≥ 58	
Smoking - n (%)	42 (11.2)	1 (1.9)	0.067	23 (14.2)	20 (7.5)	0.039^†^
Age (years) ^#^	37.0±6.5	35.7±5.9	0.177	38.5±7.2	35.8±5.7	<0.001^§^
	criteria WHO 1999		*p*	criteria WHO 2010		*p*
	With alteration	Without alteration		With alteration	Without alteration	
Obesity - n (%)	62 (25.4)	31 (15.8)	0.020	52 (24.2)	41 (18.2)	0.157^†^
	2 or more alterations 1999		*p*	2 or more alterations 2010		*P*
	Yes	No		Yes	No	
BMI (kg/m^2^)^#^	27.4±3.8	26.6±3.8	0.025	27.7±3.6	27.0±3.9	0.087^§^

* The same variables were analyzed based on TMSC without statistically significant associations (*p*>0.05).

# Mean ± standard deviation.

§ Student’s t-test

† Pearson’s chi-squared test or Fisher's exact tests

TMSC: Total Motile Sperm Count; WHO: World Health Organization

Smokers and patients with comorbidities showed a higher proportion of morphology alterations based on the 2010 WHO criteria. There was no association when these samples were categorized based on the 1999 WHO criteria or TMSC (Table 5).

In patients with volume alterations, the 1999 WHO criteria found a higher proportion of individuals with hypertension (9.5% *vs*. 3.6%, *p*=0.023) and shorter abstinence periods (Table 5). The 2010 WHO criteria and TMSC were not significantly associated with these variables.

Higher proportions of decreased sperm vitality were found in smokers and older individuals based on the 2010 WHO criteria (Table 5). The same semen samples categorized based on the 1999 WHO criteria and TMSC had no significant association.

Based on the 1999 WHO criteria, 25.4% of the obese patients had at least one alteration *versus* 15.8% of the patients with a BMI < 30 (*p*=0.02); patients with two or more alterations based on the 1999 WHO classification had significantly higher BMIs (Table 5). These associations were not found in the 2010 WHO criteria or TMSC.

## DISCUSSION

The 1999 WHO criteria for normality in semen analysis was quite stringent, and led to the categorization of men as infertile solely for their inability to conceive naturally, an element later revised in the 2010 criteria. Catanzariti *et al*. (2013) evaluated 529 semen samples from fertile and infertile patients and found that 199 (37.83%) patients were deemed normal by both criteria, 246 (46.77%) were abnormal based on the two criteria, and 82 (15.59%) were abnormal based on the 1999 criteria and normal on the 2010 WHO classification. Fifteen percent of the patients deemed abnormal based on the 1999 WHO criteria were categorized as having normal semen parameters in the 2010 classification (Catanzariti *et al*., 2013).

The samples included in this study were taken from patients seen at an assisted reproduction clinic. Approximately 84% of the samples had alterations in every parameter based on the 1999 WHO criteria; the proportion dropped to 46.8% in the 2010 criteria. When at least two clinically relevant parameters were analyzed, 61.4% had altered results in the 1999 WHO criteria against 23.5% in the 2010 classification, thereby confirming that the 1999 criteria overestimated the number of abnormal samples and cases of infertility.

Semen parameters in the 2010 WHO classification became less stringent, thus increasing the number of men with normal tests. The parameter that most influenced the difference between the classifications was morphology: 85.1% of altered samples based on the 1999 WHO criteria were deemed normal based on the 2010 criteria, along with vitality (56.3%) and motility a + b (51.3%). Only 0.6% had alterations in total concentration. Although morphology was the parameter with the greatest difference between classifications, it is not the most important element associated with reproductive outcomes. A study that evaluated 856 intrauterine insemination (IUI) cycles found no significant difference in the pregnancy rates of patients with a morphology score smaller or larger than 4% (17.3% *versus* 16.7%), suggesting that alterations in morphology should not be used in isolation as an indicator to refer patients to in vitro fertilization (IVF) (Deveneau *et al*., 2014).

Erdem *et al*. (2016) found no impact from morphology in the live birth rates of couples with unexplained infertility treated with IUI, although higher live birth rates were seen in couples with male subfertility when more than 4.5% of the spermatozoa had normal morphology.

A recent meta-analysis (Wang *et al*., 2019) suggested that varicocelectomy results in a significantly improved not only in TMSC but also in spontaneous pregnancy rate. This improvement is greater in patients with mildly or moderately decreased TMSC. Hamilton *et al*. (2015) evaluated 1177 patients with male infertility and unexplained infertility and categorized the semen samples based on the guidelines of the 2010 WHO criteria and TMSC. TMSC greater than 20 x 10^6^ was deemed normal. When the WHO criteria were used, 76% of the patients were rated as infertile, while in the evaluation based on TMSC 60% were deemed infertile.

The patients in our population were compared based on three criteria (1999 WHO, 2010 WHO, and TMSC); 84.1% had an alteration based on the 1999 WHO criteria; 46.8% based on the 2010 WHO classification; and 41.9% based on TMSC. Analysis of potential associations between alterations found that none of the parameters (concentration, motility, morphology, volume, and vitality) was significantly associated when TMSC alterations were compared to alterations identified based on the 1999 and 2010 WHO criteria.

Of the 200 samples with alterations based on TMCS, 96% had at least two alterations based on the 1999 WHO criteria against 54% in the 2010 criteria. On the other hand, of the 277 samples considered normal based on TMSC, 36.5% had more than two alterations based on the 1999 WHO criteria and only 1.4% had more than two alterations based on the 2010 WHO criteria. Since morphology is not considered in TMSC, further studies are needed to compare semen ratings and correlate the findings with natural conception and pregnancy rates in IUI.

This study showed that environmental factors, lifestyle, and chronic diseases worsen semen quality (vitality, morphology, volume), and that aging deteriorates motility and vitality. Other authors have published similar results (Du Plessis *et al*., 2010; Jurewicz *et al*., 2014; Kaya *et al*., 2020; Lingappa *et al*., 2015). The results published by Borges deserve attention. Over a period of ten years, the semen quality of patients undergoing infertility treatments showed significant decreases in concentration and percentage of normal forms, thus supporting the finding that lifestyle and environmental factors might alter male fertility.

Our study showed that in the period ranging from 1999 to 2010 the parameters became more rigid, which thus decreased the number of individuals categorized as infertile or subfertile. Normal TMSC samples correlate better with 2010 WHO criteria. The importance of sperm morphology in semen analysis and the definitions of normal and clinical outcomes need to be better studied.
